# Assessment of genetic variation in *Apis mellifera jemenitica* (Hymenoptera: Apidae) based on mitochondrial Cytochrome Oxidase Subunit II and III

This article has been retracted.

**DOI:** 10.1371/journal.pone.0265454

**Published:** 2022-03-31

**Authors:** Yehya Alattal, Ahmad Algamdi

**Affiliations:** Department of Plant Protection, Chair of Engineer Abdullah Ahmad Bagshan for Bee Research, College of Food and Agriculture Sciences, King Saud University, Riyadh, Saudi Arabia; King Khalid University, SAUDI ARABIA

## Abstract

Morphometric and genetic characterization of many *Apis mellifera* subspecies are well-documented. *A*. *m*. *jemenetica occurs* naturally in Africa and Asia. In this study, genetic variation of mitochondrial Cytochrome Oxidase II (*COII*) and III (*COIII*) were analysed in 133 specimens of the endemic honeybee colonies within Saudi Arabia. The *COII* gene sequence length was 684 bp comprising nine synonymous (1.3%) and two non-synonymous single nucleotide polymorphisms (SNPs) (0.87%). Five variants of *COII* were not previously documented, one variant (MT755968) showed an extra restriction site when subjected to type II restriction endonuclease from *Arthrobacter protophormiae* (*Apol*) or to *Haemophilus influenzae* Rf (*Hinf1*). Changes in *COII* sequence separated samples into three haplogroups. Whereas, *COIII* gene sequence length was 780 bp, including 18 synonymous and five non-synonymous SNPs. Furthermore, variation in *COII* sequence was more informative based on restriction profiles and on amino acid changes compared with *COIII* gene sequence. Variants of *COIII* showed identical restriction sites when subjected to type II restriction endonuclease from *Deinococcus radiophilus* (*DraI*), and revealed high similarity to African subspecies. Results of this study are very useful in understanding genetic diversity and characterization of *A*. *mellifera* subspecies.

## Introduction

*Apis mellifera jemenitica* spreads naturally over large geographical areas in Asia and Africa [1]. It occurs naturally in the Arabian Peninsula, Sudan, Eretria, Chad, Niger, Kenya, Tanzania, Nigeria, Niger and Ethiopia with very diverse environmental extremes [2–4]. This may imply high morphometric and genetic variations among different population of *A*. *m*. *jemenitica*. The Asian and African populations, which are isolated by the Red Sea, are very obvious example for such variation [1,5]. Although the origin of *A*. *mellifera* is still under intensive debate by many scientists, more support was recently given to an Asian (West Asian) origin [6–11]. Phylogenetic analysis based on genomic protein-coding regions sets *A*. *m*. *jemenitica* and nearby subspecies at the most basal branch of evolution [6]. In the last two decades several articles discussed the characterization of the Asian *A*. *m*. *jemenitica* [12–20]. Based on morphometric traits, Alghamdi et al (2012) reported three distinctive sub-populations of *A*. *m*. *jemenitica* from Saudi Arabia, and found significant variation compared with the African *A*. *m*. *jemenitica* populations [12]. Morphometric variation would not be unexpected among other *A*. *m*. *jemenitica* populations within Africa as well [21]. Worldwide, Ilyasove et al [13] listed 33 *A*. *mellifera* subspecies being identified based on morphometry and were assigned to five different lineages (African (A); Western Europe (M); South-Eastern Europe (C) Middle East (O) and (Y) Ethiopia). Lately Mitochondrial DNA (*mt*DNA) markers are being regularly used to characterize and investigate evolutionary relationships within *A*. *mellifera*. *mt*DNA evolves faster and it contains regions with variable evolutionary rates that is useful in addressing question in many subspecies [14,15,22,23]. COI-COII intergenic fragment is the most widely used non-coding region revealing different sequence lengths (Presence/Absence of P and Q) and number of restriction sites when subjected to type II restriction endonuclease from *Deinococcus radiophilus* (*DraI*) [10,16–20]. Using COI-COII intergenic region, *A*. *m*. *jemenitica* colonies from Saudi Arabia were identified as members of the Z sub-lineage (Previously O lineage) similar to *A*. *m*. *syriaca* and *A*. *m*. *lamarckii* [24,25]. This intergenic region is highly variable and may overcome some endemic variation among populations. Ultimately investigating variation within protein coding *mt*DNA genes is highly supportive. In this study we analyse and discuss sequence variation in *COII* and *COIII* genes for 133 non-migratory *A*. *m*. *jemenitica* samples from Saudi Arabia.

## Materials and methods

Samples of non-migratory *A*. *m*. *jemenitica* colonies (Number of samples = 133) of Saudi Arabia were collected (Makkah (n = 20); Madinah (n = 17); Taif (n = 14); Jazan (n = 16); Najran (n = 14); Tabuk (n = 18); Albaha (n = 15); Asir (n = 19)) and were then preserved in 96% Ethanol. Each sample consisted of 15 workers. All colonies were morphometrically confirmed as *A*. *m*. *jemenitica* according to standard methods [18]. For *mt*DNA analyses, DNA was extracted from one worker/colony using Qiagen extraction Kit (Cat No./ID: 69506). Extracted DNA was then sequenced by BGI (Hong Kong, China). Raw data cleaning was performed using SOAPnuke v1.5.6 (parameters -n 0.05 -l 20 -q 0.2 –G–Q 2) [26]. Filtration started with adaptor trimming (sequences with adapter mapping %>50 was removed). Next, low quality reads (Q20<50%) were removed. Finally, contiguous reads with more than 2% N bases were removed. Clean *mt*DNA reads were mapped and annotated against a reference mitogenome of *A*. *m*. *jemenitica* for a sample collected from Yemen in 1980s (GeneBank: MN714161). Mapping was performed in Geneious Prime 2020.1.2 (Biomatters Ltd., Auckland, New Zealand). Sequences of *COII* and *COIII* for each sample were then extracted in fasta format and imported to BioEdit v7.2.5 [27] for alignment with *COII* and *COIII* mtDNA sequences of other *A*. *mellifera* subspecies. *COII* and *COIII* sequences were also subjected to two restriction enzymes each*; Apol* and *Hinf*I (for COII) and *Dra*I (for *COIII*). Phylogenetic tree was constructed using Maximum Composite Likelihood method and tested over1000 bootstrap replicates [28], evolutionary distances were calculated in MEGA7 [29]. Nonsynonymous SNPs and changes on amino acid composition were also explored. Sequences were additionally analysed with Basic Local Alignment Search Tool (BLAST), then previously undocumented variants were uploaded into the Genbank.

## Results

The *COII* gene sequence length was 684bp, composed of 80.6% AT and 16.4% GC. Nine loci were polymorphic (1.3%) (Table 1) and revealed changes of two amino acids (0.87%) (Table 2). Five variants of *COII* gene sequences among *A*. *m*. *jemenitica* within Saudi Arabia were previously un-documented (Table 1). Variant-6 (MT755968: n = 4 (~3%)) revealed the highest number of nucleotide variation (Seven Nucleotides) (Table 1) and revealed ten restriction sites with *Apol* and four sited for *Hinf*1 compared with nine and three sites respectively for all other samples (Table 3). Most *COII* sequence variants (95.5%) are similar to reference sequences affiliated with the African lineage A (Table 3). However two variants (MT755968: n = 4 (~3%) and MT755970) showed an extra digestion sites for each restriction enzyme and clustered with another subspecies lineage. Table three shows variation in amino acid composition among different variants. Variant number three (MT755972) had amino acid changes on codon 93 (Valine to Isoleucine), >90% of the colonies of this variant belongs to Tabuk and Almadinah regions in the northern part of Saudi Arabia. While all colonies of variant number six had the same amino acid changes on codon 69. Interestingly Changes in amino acid compositions separated our samples into three haplogroups, Haplogroup one resembling 105 samples demonstrated identical amino acid sequence with other subspecies of the African lineage, Haplogroup two and three share similarity with subspecies from the lineage M and C respectively concerning this region. Phylogenetic tree including all *COII*-variants based on 133 samples and six other reference haplotypes using Maximum Likelihood method demonstrated that most samples clustered with *A*. *m*. *jemenitica*, *A*. *m*. *lamarckii* and *A*. *m*. *syriaca*, some samples (Variant six) clustered very close to *A*. *m*. *mellifera* (Fig 1). The *COIII* gene sequence length was 780bp, composed of 82.4% AT and 17.6% GC. Polymorphic loci were 18 (2.6%) (Table 4) resulted in five amino acids variants (1.92%) (Table 5). Nine variants were previously undocumented and were uploaded in the Genbank (Table 6). Variant number nine (MT769261: n = 4 (~3%)) revealed the highest nucleotide variation (11 nucleotides) (Table 4). *DraI* restriction profile was similar for all *COIII* Variants and were most similar to African subspecies with two restriction sites (Table 6). *COIII*–Variant number nine *(*MT769261*)* and Variant number six (MT769259) had two amino acid changes which were similar in *A*. *m*. *mellifera (*KY926884*)*. Phylogenetic tree using ML methods showed that most samples clustered with *A*. *m*. *jemenitica*, *A*. *m*. *lamarckii* and *A*. *m*. *syriaca*, however (Variant nine) clustered with *A*. *m*. *mellifera* (Fig 2).

**Fig 1:** Phylogenetic analysis for *COII* sequence variation in the study samples and seven other sequences for seven reference honeybee subspecies, using Maximum Likelihood method. Pairwise distances were estimated using the Maximum Composite Likelihood (MCL) approach, and then selecting the topology with superior log likelihood value. There were a total of 687 positions in the final dataset. Evolutionary analyses were conducted in MEGA7.

**Fig 2:** Phylogenetic tree for *COIII* sequence variation in the study samples and seven other sequences for seven reference honeybee subspecies, using the Maximum Likelihood method. Distances were estimated using the Maximum Composite Likelihood (MCL) approach, and then selecting the topology with superior log likelihood value. There were a total of 781 positions in the final dataset. Evolutionary analyses were conducted in MEGA7.

**Table 1:** Sequence variations in *COII* gene among *A*. *m*. *jemenitica* samples from Saudi Arabia. *The number of the nucleotide at the sequence resembles the position where variation took place.

Variant	Accession No.	Position of Variation											
		21	78	96	150	163	169	205	277	366	393	444	525
I	MT755967	T	T	C	T	C	T	G	G	T	C	C	T
II	MT755968	**C**	T	**T**	**C**	**T**	**C**	**A**	G	**A**	C	C	T
III	MT755969	T	**C**	C	T	C	T	G	G	T	C	C	T
IV	MT755970	T	T	C	T	C	T	**A**	G	A	C	C	T
V	(KY926882)	T	T	C	T	C	T	G	G	A	C	C	T
VI	MT755972	T	T	C	T	C	T	G	**A**	A	C	C	T
*A m jemenitica (Mn714161)*		T	T	C	T	C	T	G	G	T	C	C	T
*Am lamarckii (KY464958)*		T	T	C	T	C	T	G	G	A	T	C	T
*A m syriaca (KP163643)*		T	T	C	T	C	T	G	G	A	T	C	T
*A m intermissa (KM458618)*		**C**	T	C	T	T	T	G	G	A	T	T	C
*A m simensis (MN585108)*		T	T	C	T	T	T	G	G	A	T	T	C
*A m mellifera (KY926882)*		**C**	T	C	T	T	T	G	A	A	C	T	T

**Table 2:** Amino acid variations in *COII* gene among different haplotypes and six other reference subspecies resembling two lineages. *The number of the codon resembles the position of variation.

Haplogroup	Haplotype (distribution percent in the cluster)	No. of colonies	Codon No.		
			69	93	211
			Amino acid symbol*		
I	Haplotype-1 (5.2) (MT755967); Haplotype-1 (72.5) KY926882); Haplotype-4 (1.5) MT755969)	105	V	V	V
II	Haplotype-3 (17.3) MT755972)	24 >90% Madinah +Tabuk	V	I	V
III	Haplotype-5 (0.7) MT755970); Haplotype-6 (3) MT755968)	4 Special variant	I	**V**	V
*A m jemenitica (*MN714161*); A*. *m lamarckii (*KY464958*); A m intermissa (*KM458618*);* *A m simensis (*MN585108*)*; *A m syriaca (*KP163643*)*; *A m capensis (*KX870183*)*			V	V	V
*A m meda (*KY464957*)*, *A m caucasica (*MN714160.1*) A m carnica (*MN250878.1*);*			I	V	V
*A m ligustica (*AP018435.1*)*			I	V	I
*A m mellifera (*KY926884*)*			V	I	V

*V = Valine; I = Isoleucine.

**Table 3:** Haplotypes’ accession numbers based on *COII* gene Sequences, frequency within whole population and number of colonies in each region besides restriction map of haplotype sequences using restriction endonuclease from *Arthrobacter protophormiae* (*Apo*l) or to *Haemophilus influenzae* Rf (*Hinf*1).

Subspecies / Haplotype Accession No.		Freq. (%)	Distribution of colonies in sampling areas								Restriction map	
			Makkah	Madinah	Taif	Jazan	Najran	Tabuk	Albaha	Asir		
											*Apo*l	*Hinf*1
*A.* *m*. *jemenitica* *B.* (Saudi Arabia)	(KY926882)	72.5	16	4	12	12	12	10	15	15	6, 43, 152, 252, 341, 356, 547, 570,594 (9 positions)	38, 362, 635 (3 positions)
	MT755972	17.3	1	12	-	2		8	-	-		
	MT755967	5.2	**2**	**1**	**-**	**-**	**-**	**-**	**-**	**4**		
	MT755969	1.5	-	-	2	-		-	-	-		
	MT755970	0.7	1	-	-	-		-	-	-		
	MT755968	3.0	-	-	--	2	2	-	-	-	6, 43, 152, 160, 252, 341, 356, 547, 570, 594 (10 positions)	18, 38, 362, 635 (4 positions)
*A*. *m jemenitica* (Yemen) *(*MN714161); *A*. *m syriaca* (Syria) (KP163643)*; A*. *m lamarckii* (Egypt) *(*KY464958)											6, 43, 152, 252, 341, 356, 547, 570,594 (9 positions)	38, 362, 635 (3 positions)
*A m meda (*KY464957*)*, *A m caucasica (*MN714160.1, *A*. *m mellifera* (Germany) KY926884											6, 43, 152, 160, 252, 341, 356, 547, 570, 594 (10 positions)	18, 38, 362, 635 (4 positions)
*A*. *m simensis* (Ethiopia) MN585108											6, 43, 152, 160, 252, 341, 356 441, 547, 570, 594 (11 positions)	38, 362, 635 (3 positions)
*A*. *m intermissa* (Algeria) KM458618 *A*. *m capensis* (South Africa) KX870183											6, 43, 152, 160, 252, 341, 356, 441, 547, 570,594 (11 positions)	18, 38, 362, 635 (4 positions)

**Table 4:** Sequence variations in *COIII* gene among *A*. *m*. *jemenitica* samples from Saudi Arabia. *The number of the nucleotide at the sequence resembles the position where variation took place.

Variant	Accession No.															Position of Variation																				
		15	63	70	91	132	141	198	228	255	303	306	336	366	370	391	399	449	453	455	499	505	540	558	561	595	622	636	639	651	652	671	675	726	735	768
I	MT769253	C	T	A	G	T	T	T	T	C	T	T	T	T	A	C	G	T	T	T	C	G	C	T	T	G	T	C	T	T	T	T	C	T	T	C
II	MT769254	.	.	.	.	.	.	.	.	.	.	.	.	.	.	.	A	.	.	.	.	.	.	.	.	.	.	.	C	.	.	.	.	.	.	.
III	MT769255	.	.	.	.	.	.	.	.	.	.	.	.	.	.	.	A	.	.	.	.	.	.	.	.	.	.	.	C	.	.	C	.	.	.	.
IV	MT769262	.	.	.	.	.	.	.	.	.	.	.	.	.	.	.	A	.	.	.	.	.	.	.	.	.	.	.	.	.	.	.	.	.	.	.
V	MT769257	.	.	.	.	.	.	.	.	.	.	.	.	.	.	.	A	.	.	.	.	A	.	.	.	.	.	.	C	.	.	.	.	.	.	.
VI	MT769258	T	.	.	.	.	.	.	.	.	.	.	.	.	.	.	A	.	.	.	.	.	.	.	.	.	C	.	C	.	.	.	.	.	.	.
VII	MT769259	.	.	.	.	.	.	.	.	.	.	.	.	.	.	.	A	.	.	.	.	.	.	.	.	.	C	.	C	.	.	.	.	.	.	.
VIII	MT769260	.	.	.	.	.	.	.	.	T	.	.	.	.	.	.	A	.	.	C	.	.	.	.	.	.	.	.	C	.	.	.	.	.	.	.
IX	MT769261	.	C	.	A	.	.	C	.	T	.	C	.	C	G	.	A	.	C	.	.	.	.	C	.	.	.	.	.	C	.	.	T	.	.	.
*A m jemenitica (Mn714161)*		.	.	.	.	.	.	.	.	T	.	.	.	.	.	.	A	.	.	.	.	.	.	.	.	.	.	.	C	.	.	.	.	.	.	.
*Am lamarckii (KY464958)*		.	.	.	.	.	.	.	.	T	.	.	.	.	.	.	A	.	.	.	.	.	.	.	.	.	.	.	C	.	.	.	.	.	.	.
*A m syriaca (KP163643)*		.	.	.	.	.	.	.	.	T	.	.	.	.	.	.	A	.	.	.	.	.	.	.	.	.	.	.	C	C	.	.	.	.	.	.
*A m intermissa (KM458618)*		.	.	.	.	A	.	.	.	.	.	.	.	.	G	.	A	.	.	.	T	.	T	.	.	.	.	.	T	C	C	.	T	.	C	.
*A m simensis (MN585108)*		.	.	T	.	A	.	.	C	T	C	.	C	.	G	.	A	.	.	.	.	.	.	.	C	.	.		T	.	.	.	T	.	C	T
*A m mellifera (KY926882)*		T	.	.	A	.	A	.	.	T	.	.	.	C	G	T	A	C	.	.	.	.	.	.	.	A	.	A	.	C	.	.	T	C	.	T

**Table 5:** Amino acid variations in *COIII* gene among different haplotypes and six other reference subspecies resembling two lineages. *The number of the codon resembles the position of variation.

Amino acid variant	Haplotype (distribution percent in the cluster)	No. of colonies	Codon No.											
			24	31	44	71	119	124	150	152	163	169	199	224
			Amino acid symbol*											
I	MT769254; MT769258; MT769253; MT769262	125	I	V	F	T	D	N	L	I	S	G	A	I
II	MT769259	2	I	V	F	T	D	N	L	**T**	S	G	A	I
III	MT769255	1	I	V	F	T	D	N	L	I	S	G	A	**T**
IV	MT769257	1	I	V	F	T	D	N	L	I	S	**R**	A	I
V	MT769261, MT769259	4	I	**I**	F	T	D	**D**	L	I	S	G	A	I
*A m jemenitica (MN714161); A*. *m lamarckii (KY464958); A m syriaca (KP163643)*;			I	V	F	T	D	N	L	I	S	N	A	I
*A m simensis (MN585108)*; *A m capensis (KX870183)*			L	V	L	T	D	D	L	I	S	G	A	I
*A m intermissa (KM458618);*			I	V	L	T	D	D	L	I	S	G	A	I
*A m meda (KY464957)*, *A m caucasica (MN714160*.*1)*			I	V	L	T	N	N	L	I	L	G	A	I
*A m ligustica (AP018435*.*1;) A m carnica (MN250878*.*1);*			I	V	L	S	N	N	L	I	L	G	A	I
*A m mellifera (KY926884)*			I	I	F	T	D	D	S	I	S	G	T	I

*I = Isoleucine; V = Valine; F = Pheneyalanine; N = Asparagine; G = Glycine; T = Threonine; D = Aspartate.

**Table 6:** Haplotypes’ accession numbers based on *COIII* gene sequences, frequency within whole population and number of colonies in each region besides restriction map of haplotype sequences using *Dra*I.

	Accession No.	Freq. (%)	Distribution of COIII Variants								Digestion fragment size
											*Dra*I
			Makkah	Madinah	Taif	Jazan	Najran	Tabuk	Albaha	Asir	234, 465
**Variant**		No. (%)									
I	MT769253	0.8	**-**	**1 (100)**	**-**	**-**	**-**	**-**	**-**	**-**	
II	MT769262	1.5	-	-	2 (100)	-	-	-	--	-	
III	MT769254	82.7	20 (18)	14 (12.7)	12 (10.9)	12 (10.9)	12 (10.9)	13 (12)	11 (10)	16 (14.6)	
IV	MT769255	0.8		1(100)							
V	MT769257	0.8	-	1 (100)	-	-	-	-	-	-	
VI	MT769258	0.8						-	1(100)		
VII	MT769259	8.3	-	-	-	2 (18.2)	-	4 (36.4)	3 (27.3)	2 (18.2)	
VIII	MT769260	1.5	-	-	-	-	-	1(0.5)	1(0.5)	-	
IX	MT769261	3.0	-	-	-	2 (0.5)	2(0.5)	-	-	-	
*A*. *m jemenitica (*MN714161)*; A*. *m syriaca* (KP163643)*; A*. *m lamarckii* (KY464958)*; A*. *m intermissa* KM458618*; A*. *m capensis (*KX870183)											234, 465
*A*. *m simensis (*MN585108)											72, 132, 234, 465
*A*. *m mellifera (*KY926882)											132, 234, 465
*A m meda (KY464957)*, *A m caucasica (MN714160*.*1) A m carnica (MN250878*.*1); A m ligustica (AP018435*.*1)*											132, 234, 465

## Discussion

*A*. *m*. *jemenitica* shows high morphometric and genetic diversity and is well adapted within its distribution range [1,2,12,14,15,30]. Most publication concerned with genetic variation and phylogenetic relationship among and within *A*. *mellifera* subspecies used *mt*DNA sequences [10,14–20,31]. In this study, analyses based on *COII* and *COIII* gene sequences confirmed previous results using other *mt*DNA genes, asserting that most of the Saudi samples cluster with the *A*. *m*. *lamarckii*, *A*. *m*. *jemenitica* and *A*. *m*. *syriaca* reference samples, which resemble the African Sub lineage Z [12,14,15]. However few samples cluster with other lineages (C or O for example) or with another African sub-lineage demonstrating significant divergence from the common group. *COIII* sequences exhibited twice the variability that occurs within *COII*, furthermore variation in *COII* sequence was more informative based on restriction profile and amino acid changes compared with *COIII*. Variation in *COII* can be diagnostic for most of Almadinah and Tabuk samples (Variants MT755972) which spreads at the border line of the natural distribution range of the Syrian Honeybee *A*. *m*. *syriaca* ([1].). Apparently, ~60% of the samples from the north are restricted to the *COII*-variant six (COII-MT755972: 17.3%), which could be unique in their localities. Restriction profiles of *COII* sequences using *Apo*1 and/or *Hinf*1 demonstrated consistency with subspecies lineage grouping based on sequence variation and phylogenetic trees (Table 3), and could be used in the future in such analyses. Variation in *COIII* sequences is also unique for the variant (MT755968), which is uncommon variant found near the border of Yemen in the south, the samples resembling this variant was collected from two apiaries located about 2000m above sea level, and two other Apiaries from Najran, these four samples may be very similar to *A*. *m*. *jemenitica*. Yet, neither the presence of heterogenous groups, nor the impact of an exotic subspecies can be excluded. Although most variation in *COII* and *COIII* sequences were inconsequential and has no impact on protein structure and function, some variants had nonsynonymous SNPs and their impact on protein function should be discussed. Although reference sequences for mitochondrial genes including *COII* and *COIII* genes from the Genbank are not abundant and are available for few subspecies only, which may hinder real variability comparison in those populations and comprehensive evolutionary analysis, *A*. *m*. *lamarckii* and *A*. *m*. *syriaca* are apparently the closest to *A*. *m*. *jemenitica*, and essentially resembling the same lineage. However, based on morphometric reference data (14), it is clear that African and Asian population of *A*. *m*. *jemenitca* are closer to each other’s than to *A*. *m*. *lamarckii* and *A*. *m*. *syriaca*, which may indicate and adaptive evolution in either population. The results of this study are very useful in characterization of Saudi Arabia Honeybee, *A*. *m*. *jemenitica*.
